The article "Dual-phenotype hepatocellular carcinoma: correlation of MRI features with other primary hepatocellular carcinoma and differential diagnosis" was retracted in 2024. Reason: duplicate publication.

# Dual-phenotype hepatocellular carcinoma: correlation of MRI features with other primary hepatocellular carcinoma and differential diagnosis

**DOI:** 10.3389/fonc.2023.1253873

**Published:** 2024-01-11

**Authors:** Liqing Zhang, Jing Chen, Xufeng Lai, Xiaoqian Zhang, Jianfeng Xu

**Affiliations:** ^1^ Department of Radiology, Affiliated Hangzhou First People's Hospital, School of Medicine, Westlake University, Hangzhou, China; ^2^ Department of Radiology, Shulan (Hangzhou) Hospital Affiliated to Zhejiang Shuren University Shulan International Medical College, Hangzhou, China

**Keywords:** hepatocellular carcinoma, dual-phenotype hepatocellular carcinoma, intrahepatic cholangiocarcinoma, magnetic resonance imaging, diagnosis

## Abstract

**Objectives:**

Dual-phenotype hepatocellular carcinoma (DPHCC) is a rare subtype of hepatocellular carcinoma characterized by high invasiveness and a poor prognosis. The study aimed to compare clinical and magnetic resonance imaging (MRI) features of DPHCC with that of non-DPHCC and intrahepatic cholangiocarcinoma (ICC), exploring the most valuable features for diagnosing DPHCC.

**Methods:**

A total of 208 cases of primary liver cancer, comprising 27 DPHCC, 113 non-DPHCC, and 68 ICC, who undergone gadoxetic acid–enhanced MRI, were enrolled in this study. The clinicopathologic and MRI features of all cases were summarized and analyzed. Univariate and multivariate logistic regression analyses were conducted to identify the predictors. Kaplan–Meier survival analysis was used to evaluate the 1-year and 2-year disease-free survival (DFS) and overall survival (OS) rates in the cohorts.

**Results:**

In the multivariate analysis, the absence of tumor capsule (*P =* 0.046; OR = 9.777), persistent enhancement (*P =* 0.006; OR = 46.941), arterial rim enhancement (*P =* 0.011; OR = 38.211), and target sign on DWI image (*P =* 0.021; OR = 30.566) were identified as independently significant factors for distinguishing DPHCC from non-DPHCC. Serum alpha-fetoprotein (AFP) >20 μg/L (*P =* 0.036; OR = 67.097) and hepatitis B virus (HBV) positive (*P =* 0.020; OR = 153.633) were independent significant factors for predicting DPHCC compared to ICC. The 1-year and 2-year DFS rates for patients in the DPHCC group were 65% and 50%, respectively, whereas those for the non-DPHCC group were 80% and 60% and for the ICC group were 50% and 29%, respectively. The 1-year and 2-year OS rates for patients in the DPHCC group were 74% and 60%, respectively, whereas those for the non-DPHCC group were 87% and 70% and for the ICC group were 55% and 37%, respectively. Kaplan–Meier survival analysis revealed significant differences in the 1-year and 2-year OS rates between the DPHCC and non-DPHCC groups (*P* = 0.030 and 0.027) as well as between the DPHCC and ICC groups (*P* = 0.029 and 0.016).

The article "Dual-phenotype hepatocellular carcinoma: correlation of MRI features with other primary hepatocellular carcinoma and differential diagnosis" was retracted in 2024. Reason: duplicate publication.

**Conclusion:**

In multi-parameter MRI, combining the assessment of the absence of tumor capsule, persistent enhancement, arterial rim enhancement, and target sign on DWI image with clinical data such as AFP >20 μg/L and HBV status may support in the diagnosis of DPHCC and differentiation from non-DPHCC and ICC. Accurate preoperative diagnosis facilitates the selection of personalized treatment options.

## Introduction

Primary liver cancer ranks as the sixth most common malignancy and the third leading cause of cancer-related death in the world (1). Primary liver cancer is categorized into three types by the World Health Organization: hepatocellular carcinoma (HCC), intrahepatic cholangiocarcinoma (ICC), and combined HCC-cholangiocarcinoma (cHCC-CCA) (2), with HCC accounting for 90% (3). Significant advancements in therapeutic methods have been achieved for both the early and advanced stages of HCC in recent decades. However, the recurrence rate remains high, and the long-term outcomes remain unsatisfactory (4). Although certain biomarkers (5, 6) and tumor staging systems (7, 8) can predict the prognosis to some extent, there are significant individual variations in HCC prognoses that cannot be accurately predicted by these methods.

Dual-phenotype HCC (DPHCC), a newly reported subtype of HCC in 2011, accounts for approximately 10% of HCC cases (9). According to the Chinese Guidelines for Standardized Pathological Diagnosis of Primary Liver Cancer (2015 Edition) (10), DPHCC is characterized by the histopathological appearance of typical HCC, along with the expression of HCC markers (e.g., hepatocyte paraffin 1 (HepPar-1), polyclonal carcinoembryonic antigen (pCEA), and glypican 3 (GLY 3)) and ICC markers (e.g., cytokeratin 19 (CK19) and mucin 1 (MUC-1)), indicating dual biological behaviors of HCC and ICC. Studies (11–14) had demonstrated that the expression of CK19 can promote cell proliferation, invasiveness, and metastasis in DPHCC, resulting in a poor prognosis. Therefore, DPHCC has a higher degree of malignancy and poor prognosis, requiring early diagnosis, and effective treatment is very important.

The diagnosis of this DPHCC primarily relies on invasive immunohistochemical detection, which can potentially lead to complications. Preoperative magnetic resonance imaging (MRI) diagnosis has emerged as a crucial noninvasive method for diagnosing liver cancer, enabling the avoidance of biopsies and the prevention of serious complications. MRI provides extensive diagnostic information through multi-parameter and multi-sequence imaging. In recent years, with the rapid development of artificial intelligence, a few studies (15, 16) had applied radiomics to preoperatively diagnose DPHCC. However, the limited sample size and single-center data in some study may hinder the generalization of the model.

The article "Dual-phenotype hepatocellular carcinoma: correlation of MRI features with other primary hepatocellular carcinoma and differential diagnosis" was retracted in 2024. Reason: duplicate publication.

Few studies had focused on the imaging features of DPHCC, particularly regarding the qualitative and quantitative characteristics of MRI imaging. This study aimed to identify MRI features and clinical factors that can help in the early diagnosis of DPHCC, potentially leading to improved treatment strategies and patient outcomes.

## Materials and methods

### Patients

This retrospective study was approved by the Medical Ethics Committees of Shulan (Hangzhou) Hospital, and the requirement for informed consent was waived. The data were collected from 208 patients who had pathologically confirmed between January 2016 and June 2020. The clinical and pathological data contained gender, age, laboratory examinations, microvascular invasion (MVI), and metastasis. The inclusion criteria were as follows (1): Patients who underwent surgery or transplantation and were pathologically confirmed to have primary liver cancer, including DPHCC and non-DPHCC (defined as CK7- and CK19-negative HCC) (2); contrast-enhanced MRI was performed within 2 weeks before surgery; and (3) availability of complete clinical data. The exclusion criteria were as follows (1): history of local-tumor therapy (n = 30) (2); with a history of other tumors(n = 25) (3); interval longer than 2 weeks between MRI examination and surgery (n = 9) (4); incomplete clinical data or poor MRI quality (n = 35) (4); recurrent cases (n = 36) (5); and pathologically confirmed cHCC-CCA (n = 15). The study workflow is summarized in **Figure 1**.

**Figure 1:** Flow diagram of the study.

### MRI protocols

Patients underwent a 4-h fasting period prior to MRI scanning, during which no water intake was allowed. Gadopentetate dimeglumine (Gd-DTPA) (*Magnevist*, Bayer Schering Pharma, Berlin, Germany) was administered as the contrast agent at a dose of 0.1 mmol/kg, with an injection velocity of 2 mL/s. The arterial phase, portal venous phase, and delayed phase were scanned at 18–23 s, 50–60 s, and 150–180 s after intravenous injection, respectively.

MR abdominal examinations were conducted by GE Signa HDxt 1.5-T MR apparatus (GE, Medical System, Milwaukee, USA) and Siemens Magnetom Skyra 3.0-T MR (Siemens, Healthineers, Berlin and Munich, Germany) with an abdominal eight-channel phased-array coil. Conventional MRI examination sequences included the following: respiratory gating T2-weighted fat-suppressed sequence (T2WI), T1-weighted in-phase and opposed-phase (IP/OP), free-breath diffusion-weighted imaging (DWI) with b-value of 0 s/mm^2^ and 800 s/mm^2^, T1-weighted fat-suppressed sequence, and three phases of enhancement. Apparent diffusion coefficient (ADC) maps were derived from the DWI sequence. Details of scanning sequences and parameters are shown in **Table 1**.

The article "Dual-phenotype hepatocellular carcinoma: correlation of MRI features with other primary hepatocellular carcinoma and differential diagnosis" was retracted in 2024. Reason: duplicate publication.

**Table 1:** Detailed parameters of different MR sequences.

Scanner	Sequence	TR (ms)	TE (ms)	Matrix	FOV (mm^2^)	Slice thickness (mm)	Gap (mm)	Number of slices	Flip angle (°)
GE Signa Hdxt 1.5T	IP/OP	6.1	4.2	224 × 224	400 × 400	5	0	68	15
	T2WI	4500	90-100	320 × 192	380 × 380	6	1.2	24	90
	DWI	10588.2	71.5	128 × 128	380 × 380	6	1	24	90
	T1WI+C	4.2	2.0	320×224	400 × 400	5	0	68	15
Siemens MAGNETOM Skyra 3.0T	IP/OP	170	1.3	320 × 256	380 × 380	5	0	76	12
	T2WI	3000	84	320 × 320	380 × 380	5	1.2	25	90
	DWI	6300	54	126 × 126	380 × 380	5	1	25	90
	T1WI+C	3.67	1.34	320 × 240	380 × 380	5	0	76	12

DWI, diffusion-weighted imaging; FOV, field of view; IP, in-phase; OP, opposed-phase; T1WI, T1-weighted imaging; T2WI, T2-weighted imaging; TE, echo time; TR, repetition time.

### Morphological features of MRI images

MRI morphological features were assessed by two abdominal radiologists (with 8 years and more than 15 years of experience) who were blinded to the pathology by using a picture archiving and communication system. If there was a discrepancy between two radiologists, then a third abdominal radiologist reviewed and reached a consensus. The following quantitative and qualitative imaging parameters were evaluated (1): tumor size (maximum diameter on the axial T2WI) (2); tumor number (3); tumor margin (smooth or irregular) (4); tumor capsule (5); hemorrhagic component (hyperintensity on T1WI images) (6); fat component (low signal intensity on in/out-phase images) (7); necrosis or cystic (high signal intensity on T2WI images without enhancement) (8); high signal ring on T2WI image, high signal ring compared to tumor parenchyma (9); enhancement pattern: i. fast-in and fast-out and ii. persistent enhancement (10); intratumor nodular enhancement (11); arterial rim enhancement (12); target sign on DWI image (b = 800 s/mm^2^) (13); ADC value; and (14) tumor–to–right erector spinae signal intensity ratio on T2WI image; the signal intensity of tumor and erector spinae at the same level was measured with the same size, with the exclusion of regions of vessels, hemorrhagic areas, and cystic lesion whenever possible. The region of interest was measured three times and averaged.

### Prognostic analysis

All of the patients were followed up as outpatients or by telephone for 1–24 months after treatment. The presence or absence of tumor was determined using enhanced computed tomography (CT) or MRI. The data cutoff was 30 June 2022.

The article "Dual-phenotype hepatocellular carcinoma: correlation of MRI features with other primary hepatocellular carcinoma and differential diagnosis" was retracted in 2024. Reason: duplicate publication.

### Statistical analysis

Statistical analysis was performed using SPSS (version 26.0) and MedCalc (version 19.1). Continuous variables were statistically analyzed by *t*-test. The Mann–Whitney U-test, chi-square test, and Fisher’s exact test were used to evaluate the univariate statistical differences among clinic characteristics and MRI parameters. The clinical and imaging features with statistically significant differences were selected. Univariate and multivariate logistic regression analyses were performed to identify independent risk factors. Kaplan–Meier survival analysis was used to assess 1-year and 2-year PFS and OS. The log-rank test was conducted to compare survival differences among the groups. *P* < 0.05 was considered to be statistically significant.

## Result

### Clinicopathological characteristics

The study comprised 27 patients with DPHCC (12 men and 15 women; mean age, 54.8 ± 10.7 years), 113 patients with non-DPHCC (104 men and 9 women; mean age, 58.2 ± 10.3 years), and 68 patients with ICC (31 men and 37 women; mean age, 59.6 ± 10.7 years). Gender was the statistical difference in the DPHCC and non-DPHCC groups (*P* = 0.000), with a higher prevalence of women in the DPHCC group. There were no significant differences in age, tumor markers, hepatitis B virus (HBV) infection, cirrhosis, MVI, and lymphatic or distant metastasis. Compared with the ICC group, there were statistical differences in alpha-fetoprotein (AFP), CA19-9, CE125, HBV infection, liver cirrhosis, MVI, and lymph node metastasis. The incidence of AFP >20 μg/L in the DPHCC group was significantly higher than that in the ICC group (*P* = 0.000), whereas the incidence rates of CA19-9 >37 kU/L and CA125 >35 kU/L in the DPHCC group were significantly lower than that in the ICC group. Furthermore, HBV positive and liver cirrhosis in the DPHCC group were more common than that in the ICC group (*P* = 0.000). The incidence rates of MIV and lymphatic and distant metastasis in the DPHCC group was lower than that in the ICC group, with a statistical significance (*P* = 0.020, 0.000). No statistical differences were observed in terms of gender, age, CEA, or distant metastasis. The clinicopathological characteristics of the three groups are summarized in **Table 2**.

**Table 2:** Comparison of clinicopathologic characteristics between the DPHCC, non- DPHCC, and ICC groups.

	DPHCC (n = 27)	Non-DPHCC (n = 113)	ICC (n = 68)	P^*^-value	P^**^-value
Gender				0.000	0.920
Male	12 (44.4%)	104 (92.0%)	31 (45.6%)		
Female	15 (55.6%)	9 (8.0%)	37 (54.4%)		
Age (years)	54.8 ± 10.7	58.2 ± 10.3	59.6 ± 10.7	0.088	0.052
AFP > 20 μg/L	18 (66.7%)	60 (53.1%)	4 (5.9%)	0.202	0.000
CA19-9 > 37 kU/L	3 (11.1%)	11 (9.7%)	46 (67.6%)	1.000	0.000
CEA > 5 μg/L	5 (18.5%)	11 (9.7%)	25 (36.8%)	0.341	0.084
CA125 > 35 kU/L	4 (14.8%)	19 (16.8%)	38 (55.9%)	1.000	0.000
BCLC stage				0.318	0.426
0/A	14 (51.9%)	60 (53.1%)	34 (50.0%)		
B	10 (37.0%)	38 (33.6%)	25 (36.8%)		
C	3 (11.1%)	15 (13.3%)	9 (13.2%)		
HBV				1.000	0.000
Yes	26 (96.3%)	108 (95.6%)	10 (14.7%)		
No	1 (3.7%)	5 (4.4%)	58 (85.3%)		
Liver cirrhosis				0.297	0.000
Yes	19 (70.4%)	90 (79.6%)	9 (13.2%)		
No	8 (29.6%)	23 (20.4%)	59 (86.8%)		
MVI				0.601	0.020
Yes	5 (18.5%)	14 (12.4%)	30 (44.1%)		
No	22 (81.5%)	99 (87.6%)	38 (55.9%)		
Lymphatic metastasis				0.364	0.000
Yes	4 (14.8%)	8 (7.1%)	40 (58.8%)		
No	23 (85.2%)	105 (92.9%)	28 (41.2%)		
Distant metastasis				0.214	0.064
Yes	4 (14.8%)	5 (4.4%)	23 (33.8%)		
No	23 (85.2%)	108 (95.6%)	45 (66.2%)		

AFP, alpha-fetoprotein; BCLC, Barcelona Clinic Liver Cancer; DPHCC, dual-phenotype hepatocellular carcinoma; HBV, hepatitis B virus; ICC, intrahepatic cholangiocarcinoma; MVI, microvascular invasion; P^*^, DPHCC vs. non-DPHCC; P^**^, DPHCC vs. ICC. P < 0.05.

The article "Dual-phenotype hepatocellular carcinoma: correlation of MRI features with other primary hepatocellular carcinoma and differential diagnosis" was retracted in 2024. Reason: duplicate publication.

### Comparison of MRI features between DPHCC and Non-DPHCC and between DPHCC and ICC

Among the qualitative parameters, there were statistically significant differences in tumor margin, tumor capsule, fat component, enhancement pattern, intratumor nodular enhancement, arterial rim enhancement, target sign on DWI image, and ADC value between the DPHCC group and the non-DPHCC group. Smooth tumor margin, the presence of tumor capsule, and fat component were less in the DPHCC group, whereas persistent enhancement, intratumor nodular enhancement, arterial rim enhancement, and target sign on DWI enhancement were more common in the DPHCC group. In addition, the ADC value was lower in the DPHCC group than non-DPHCC (*P =* 0.009). Conversely, fast-in and fast-out enhancement patterns were more common in the non-DPHCC group. A typical image of DPHCC are shown in **Figure 2**.

**Figure 2:** Dual-phenotype hepatocellular carcinoma in a 46-year-old man with AFP of 1261 μg/L and positive hepatitis B virus. **(A)** The tumor showed a moderate hyperintense on T2-weighted imaging with a slightly higher signal ring compared to the surrounding tumor parenchyma. **(B)** Target sign on DWI image (b = 800 s/mm^2^). **(C)** The tumor showed a hypointensity on T1-weighted imaging. **(D)** Arterial rim enhancement. **(E, F)** Persistent enhancement.

The DPHCC group exhibited statistically significant differences in tumor size, tumor margin, enhancement pattern, intratumor nodular enhancement, and arterial rim enhancement compared with the ICC group. The tumor size in the DPHCC group was smaller than that in the ICC group, and the tumor margin was smoother. Fast-in and fast-out enhancement pattern and arterial rim enhancement were more common in the DPHCC group compared with that in the ICC group. In contrast, intratumor nodular enhancement was more common in the ICC group. No statistically significant differences were found for the remaining features. Among the quantitative parameters, the tumor diameter of the DPHCC group was smaller than that of the ICC group. In addition, the tumor–to–right erector spinal signal ratio on T2WI images was higher in the DPHCC group compared with that in the non-DPHCC group (*P* = 0.000) and was lower compared with that in the ICC group (*P* = 0.070). Quantitative and qualitative MRI features in three groups are presented in **Table 3**.

The article "Dual-phenotype hepatocellular carcinoma: correlation of MRI features with other primary hepatocellular carcinoma and differential diagnosis" was retracted in 2024. Reason: duplicate publication.

**Table 3:** Comparison of MRI features between the DPHCC, non-DPHCC, and ICC groups.

	DPHCC (n = 27)	Non-DPHCC (n = 113)	ICC (n = 68)	P^*^-value	P^**^-value
Median Tumor size (range, cm)	4.62 ± 3.02	4.76 ± 3.49	6.69 ± 3.54	0.914	0.006
Tumor number				0.570	0.071
Single	19 (70.4%)	73 (64.6%)	34 (50.0%)		
Multiple	8 (29.6%)	40 (35.4%)	34 (50.0%)		
Tumor margin				0.000	0.000
Smooth	8 (29.6%)	92 (81.4%)	1 (1.5%)		
Irregular	19 (70.4%)	21 (18.6%)	67 (98.5%)		
Tumor capsule				0.000	0.073
Yes	8 (29.6%)	82 (72.6%)	8 (11.8%)		
No	19 (70.4%)	31 (27.4%)	60 (88.2%)		
Hemorrhagic component				0.243	1.000
Yes	1 (3.7%)	16 (14.2%)	3 (4.4%)		
No	26 (96.3%)	97 (85.8%)	65 (95.6%)		
Fat component				0.000	0.166
Yes	2 (7.4%)	63 (55.8%)	15 (22.1%)		
No	25 (92.6%)	50 (44.2%)	53 (77.9%)		
Necrosis or cystic				0.787	0.311
Yes	12 (44.4%)	47 (41.6%)	21 (30.9%)		
No	15 (55.6%)	66 (58.4%)	47 (69.1%)		
High signal ring on T2WI image				0.104	0.092
Yes	6 (22.2%)	10 (8.8%)	5 (7.4%)		
No	21 (77.8%)	103 (91.2%)	63 (92.6%)		
Enhancement pattern				0.000	0.001
Fast in and fast out	8 (29.6%)	107 (94.7%)	2 (2.9%)		
Persistent reinforcement	19 (70.4%)	6 (5.3%)	66 (97.1%)		
Intratumor nodular enhancement				0.000	0.016
Yes	20 (74.1%)	5 (4.4%)	64 (94.1%)		
No	7 (25.9%)	108 (95.6%)	4 (5.9%)		
Arterial rim enhancement				0.000	0.024
Yes	20 (74.1%)	9 (8.0%)	33 (48.5%)		
No	7 (25.9%)	104 (92.0%)	35 (51.5%)		
Target sign on DWI image				0.000	0.329
Yes	21 (77.8%)	7 (6.2%)	46 (67.6%)		
No	6 (22.2%)	106 (93.8%)	22 (32.4%)		
ADC value	956.21 ± 253.41	1172.01 ± 346.26	1050.43 ± 349.04	0.009	0.157
Tumor–to–right erector spinal signal ratio on T2WI images	3.54 ± 1.76	2.22 ± 1.20	4.03 ± 2.45	0.000	0.070

ADC, apparent diffusion coefficient; DPHCC, dual-phenotype hepatocellular carcinoma; ICC, intrahepatic cholangiocarcinoma; P^*^, DPHCC vs. non-DPHCC; P^**^, DPHCC vs. ICC. P < 0.05.

The article "Dual-phenotype hepatocellular carcinoma: correlation of MRI features with other primary hepatocellular carcinoma and differential diagnosis" was retracted in 2024. Reason: duplicate publication.

### Risk factors for DPHCC diagnosis

Univariate and multivariate logistic regression analyses revealed that, in the DPHCC group versus the non-DPHCC group, the absence of the tumor capsule (*P* = 0.046; OR = 9.777), persistent enhancement (*P* = 0.006; OR = 46.941), arterial rim enhancement (*P =* 0.011; OR = 38.211), and target sign on DWI image (*P* =0.021; OR = 30.566) were the independent predictors of DPHCC (**Table 4**). Whereas, in the DPHCC group versus the ICC group, AFP> 20 μg/L (*P =* 0.036; OR = 67.097) and HBV infection (*P =* 0.020; OR = 153.633) emerged as the independent risk factors of DPHCC (**Table 5**).

**Table 4:** Univariate and multivariate logistic regression analyses of variables in predicting DPHCC between DPHCC and non-DPHCC.

	Univariate analysis		Multivariate analysis	
	*P* value	OR (95% CI)	*P* value	OR (95% CI)
Tumor margin	0.000	10.405 (4.014, 26.968)		
Absence of tumor capsule	0.000	6.282 (2.494, 15.822)	0.046	9.777 (1.037, 92.218)
Fat component	0.202	2.688 (0.588, 12.280)		
Contrast enhancement pattern	0.000	42.354 (13.204, 135.859)	0.006	46.941 (3.005, 733.275)
Nodular enhancement intratumor	0.000	61.724 (17.808, 213.873)		
Arterial rim enhancement	0.000	33.016 (11.017, 98.943)	0.011	38.211 (13.708, 99.165)
Tumor–to–right erector spinal signal ratio on T2WI image	0.000	0.547 (0.404, 0.740)		
Target sign on DWI image	0.000	53.000 (16.177, 173.636)	0.021	30.566 (1.678, 553.970)

AFP, alpha-fetoprotein; DPHCC, dual-phenotype hepatocellular carcinoma; HBV, Hepatitis B virus; ICC, intrahepatic cholangiocarcinoma.

**Table 5:** Univariate and multivariate logistic regression analyses of variables in predicting DPHCC between DPHCC and ICC.

Variables	Univariate analysis		Multivariate analysis	
	*P* value	OR (95% CI)	*P* value	OR (95% CI)
AFP > 20 μg/L	0.000	23.000 (6.282, 84.203)	0.036	67.097 (1.307, 344.311)
CEA > 5 μg/L	0.043	3.186 (1.038, 9.782)		
CA125 > 35 kU/L	0.001	7.318 (2.205, 24.289)		
CA199 > 37 kU/L	0.000	17 (4.455, 64.876)		
HBV	0.000	190.667 (21.731, 1672.936)	0.020	153.633 (2.176, 1848.946)
Liver cirrhosis	0.000	17.417 (5.312, 57.101)		
Tumor margin	0.006	20.632 (2.415, 176.285)		
Contrast enhancement pattern	0.006	10.105 (1.964, 51.992)		
Intratumor nodular enhancement	0.011	0.179 (0.047, 0.673)		
Arterial rim enhancement	0.044	2.857(1.026, 7.954)		

DPHCC, dual-phenotype hepatocellular carcinoma; HBV, hepatitis B virus; ICC, intrahepatic cholangiocarcinoma.

### Prognosis

As of June 2022, all patients (n = 208) completed follow-up for disease-free survival (DFS) and overall survival (OS). The 1-year and 2-year DFS rates for patients in the DPHCC group were 65% and 50%, respectively, whereas those for the non-DPHCC group were 80% and 60% and for the ICC group were 50% and 29%, respectively. The 1-year and 2-year OS rates for patients in the DPHCC group were 74% and 60%, respectively. Kaplan–Meier survival analysis showed there were differences in 1-year and 2-year OS between the DPHCC and non-DPHCC groups (*P* = 0.030 and 0.027), as well as between the DPHCC and ICC groups (*P* = 0.029 and 0.016) (**Figure 3**).

The article "Dual-phenotype hepatocellular carcinoma: correlation of MRI features with other primary hepatocellular carcinoma and differential diagnosis" was retracted in 2024. Reason: duplicate publication.

**Figure 3:** Kaplan–Meier survival analysis. The OS of DPHCC, non-DPHCC, and ICC.

## Discussion

DPHCC, a recently defined rare subtype of HCC, exhibits dual biological characteristics of HCC and ICC, resulting in a higher degree of malignancy and a poorer prognosis. Consequently, the preoperative noninvasive diagnosis of DPHCC holds a significant clinical value. Our results indicated that the absence of tumor capsule, persistent enhancement, arterial rim enhancement, and target sign on DWI image may serve as important features potentially predictive of DPHCC compared with that of non-DPHCC. Compared with ICC, APF >20μg/L and a history of HBV infection are the important indicators for the potential prediction of DPHCC. We speculate that DPHCC tends to resemble ICC in imaging manifestations and resembles non-DPHCC in clinical and laboratory data. Combining imaging and clinical features are of great value in the preoperative diagnosis of DPHCC.

Compared with the non-DPHCC group, only gender differed in clinicopathological features, with a higher proportion of women in the DPHCC group and a higher incidence of men in non-DPHCC group. Our previous research also identified gender as a risk factor, with a higher proportion of CK19+ HCC in women. This association may be linked to estrogen, although further investigation with larger sample sizes is needed to explore this hypothesis. Statistically significant differences were observed in tumor margin, tumor capsule, fat component, enhancement pattern, intratumor nodular enhancement, arterial rim enhancement, and the target sign on DWI image. Notable factors potentially predictive of DPHCC included the absence of tumor pseudocapsule, persistent enhancement, arterial rim enhancement, and target sign on DWI image. The formation of the pseudocapsule is assumed to result from tumor expansion and compression of the adjacent liver tissue, leading to fibrous connective tissue proliferation (17, 18). Studies have shown that the presence of pseudocapsule, especially complete tumor capsule, is associated with a favorable prognosis after tumor therapy (19, 20). In addition, without capsule of HCC is demonstrated to exhibit greater malignancy. Our study showed that the absence of tumor capsule was an independent risk factor for predicting DPHCC, which suggested more malignancy of DPHCC. In addition, the OS of the DPHCC group in our study was significantly lower than that of the non-DPHCC group. Our findings indicated that the enhancement pattern of most DPHCC was persistent rather than typical fast-in and fast-out, which resembled the imaging findings of ICC (21, 22). Our results showed no statistical difference in enhancement patterns between the DPHCC and ICC groups. The reason for this enhancement pattern may be related to the expression of tumor markers of bile duct cells (CK7 and CK19) by DPHCC. CK19 is considered a stem cell marker and is assumed to indicate the differentiation of HCC toward the biliary tract and the production of connective tissue mesenchyme within tumors (23). This component could prolong the retention time of the contrast agent, leading to a persistent enhancement pattern resembling that of ICC. Our previous study (24) found that arterial rim enhancement was an independent predictor of CK19+ HCC. In the current study, arterial rim enhancement also emerged as an independent predictor for diagnosing DPHCC, aligning with the findings of Wang et al. (25). Another study (26) demonstrated a higher incidence of arterial rim enhancement in CK19+ HCC, and there was no significant difference in target sign on DWI between CK19− and CK19+ HCC. However, our study showed target sign on DWI image as an independent predictor for diagnosing DPHCC, and the corresponding ADC value of DPHCC was lower than that of non-DPHCC and ICC. We speculate that these two features have a similar pathological basis, potentially associated with the expression of CK19. Several studies reported that these two characteristics were also independent risk factors for diagnosing small ICC (27, 28), suggesting that the similarity in pathological features contributes to the resemblance in image appearance of DPHCC. Our study included these liver cancers scanned by 1.5-T and 3.0-T MRI, and previous literatures had shown that increasing the field intensity can improve image quality, mainly improving the signal-to-noise ratio. Thus, we did not analyze the difference between different field intensity.

The article "Dual-phenotype hepatocellular carcinoma: correlation of MRI features with other primary hepatocellular carcinoma and differential diagnosis" was retracted in 2024. Reason: duplicate publication.

Multivariate regression analysis showed that, compared with the ICC group, AFP >20μg/L and HBV positive were the independent risk factors for predicting DPHCC, which is consistent with a previous study (9). This correlation may be attributed to the expression of HCC markers by DPHCC. Although MRI features were not identified as independent risk factors, our findings showed that ICC had larger tumor sizes and more irregular margins, which could be associated with a poorer prognosis for ICC. Wu et al. (29) analyzed the signal intensity ratio between lesion and liver parenchyma at each stage. They found that the intensity of the lesion and signal intensity ratio at the portal vein phase were important independent variables for the potential prediction of DPHCC, which indicated the difference in the enhancement pattern between DPHCC and non-DPHCC. In our study, we applied the tumor–to–right erector spinal signal ratio on T2WI images to reflect the changes in the T2 intensity of the tumor. The signal intensity ratio of DPHCC was between that of non-DPHCC and ICC. It may be related to the amount of water in the tumor. Further studies are needed to validate the value of this quantitative parameter with large samples. Our study achieved some independent risk factors for diagnosing DPHCC, which were mainly qualitative characteristics. There may be subjective differences in their diagnosis. More quantitative parameters and radiomics will be of future research.

Our study has been 1-year and 2-year follow-up of these three groups, revealing that the DFS and OS rates were lower in the DPHCC group compared with that in the non-DPHCC group but higher than that in the ICC group. The results of 1-year DFS and OS in the DPHCC and non-DPHCC groups aligned with those by Huang et al. (15). Currently, there were limited studies on the prognosis of DPHCC. Huang et al. performed a 1-year follow-up comparing DPHCC and non-DPHCC, which showed lower DFS and OS rates in the DPHCC group, but without a statistical difference. In our study, there were statistical differences in 1-year and 2-year DFS and OS. These disparities could be attributed to variations in the inclusion criteria between the two studies. The patients who were rolled in our study underwent surgical resection or liver transplantation. Notably, our results demonstrated a worse prognosis for ICC when compared to DPHCC. There was no study that compared the prognosis of DPHCC with that of ICC.

There were several limitations to our study. Firstly, it was a retrospective study and may have selection bias. Secondly, the sample was small, and the study was performed at a single center, requiring larger sample sizes of multi-centers to further study. Also, patients with liver-specific contrast agent were small samples too, and more patients will be collected. Thirdly, because the small sample of cHCC-CCA was not included in our study, future research should focus on this aspect.

## Conclusion

In summary, our study highlights the significance of multi-parameter MRI imaging, including the absence of tumor capsule, persistent enhancement pattern, arterial rim enhancement, and target sign on DWI image, along with clinical laboratory features such as serum AFP >20 μg/L and HBV infection, in the diagnosis and differential diagnosis of DPHCC. These features potentially help in the early and accurate diagnosis of DPHCC and improve treatment strategies and patient outcomes.

The article "Dual-phenotype hepatocellular carcinoma: correlation of MRI features with other primary hepatocellular carcinoma and differential diagnosis" was retracted in 2024. Reason: duplicate publication.

## Data availability statement

The raw data supporting the conclusions of this article will be made available by the authors, without undue reservation.

## Ethics statement

The studies involving humans were approved by Shulan (Hangzhou) Hospital Affiliated to Zhejiang Shuren University Shulan International Medical College. The studies were conducted in accordance with the local legislation and institutional requirements. Written informed consent for participation was not required from the participants or the participants’ legal guardians/next of kin in accordance with the national legislation and institutional requirements. Written informed consent for participation was not required for this study in accordance with the national legislation and the institutional requirements.

## Author contributions

LZ: Data curation, Funding acquisition, Methodology, Writing – original draft. JC: Formal analysis, Investigation, Data curation, Writing – review & editing. XL: Formal analysis, Investigation, Methodology, Supervision, Writing – original draft. XZ: Investigation, Methodology, Software, Writing – original draft. JX: Project administration, Resources, Validation, Visualization, Writing – review & editing.

## References

[1] SungHFerlayJSiegelRLLaversanneMSoerjomataramIJemalA. Global cancer statistics 2020: GLOBOCAN estimates of incidence and mortality worldwide for 36 cancers in 185 countries. CA A Cancer J Clin (2021) 71:209–49. doi: 10.3322/caac.21660 33538338

[2] LaursenL. A preventable cancer. Nature (2014) 516:S2–3. doi: 10.1038/516S2a 25470197

[3] XiaCDongXLiHCaoMSunDHeS. Cancer statistics in China and United States, 2022: profiles, trends, and determinants. Chin Med J (Engl) (2022) 135:584–90. doi: 10.1097/CM9.0000000000002108 PMC892042535143424

[4] SugawaraYHibiT. Surgical treatment of hepatocellular carcinoma. Biosci Trends (2021) 15:138–41. doi: 10.5582/bst.2021.01094 33746184

[5] GallePRFoersterFKudoMChanSLLlovetJMQinS. Biology and significance of alpha-fetoprotein in hepatocellular carcinoma. Liver Int (2019) 39:2214–29. doi: 10.1111/liv.14223 31436873

[6] FengHLiBLiZWeiQRenL. PIVKA-II serves as a potential biomarker that complements AFP for the diagnosis of hepatocellular carcinoma. BMC Cancer (2021) 21:401. doi: 10.1186/s12885-021-08138-3 33849479 PMC8045263

[7] BhandareMSPatkarSShettyNPolnayaAKulkarniSDusaneRR. Liver resection for HCC outside the BCLC criteria. Langenbecks Arch Surg (2018) 403:37–44. doi: 10.1007/s00423-017-1640-3 29199380

The article "Dual-phenotype hepatocellular carcinoma: correlation of MRI features with other primary hepatocellular carcinoma and differential diagnosis" was retracted in 2024. Reason: duplicate publication.

[8] VitaleABurraPFrigoACTrevisaniFFarinatiFSpolveratoG. Survival benefit of liver resection for patients with hepatocellular carcinoma across different Barcelona Clinic Liver Cancer stages: a multicentre study. J Hepatol (2015) 62:617–24. doi: 10.1016/j.jhep.2014.10.037 25450706

[9] LuX-YXiTLauW-YDongHZhuZShenF. Hepatocellular carcinoma expressing cholangiocyte phenotype is a novel subtype with highly aggressive behavior. Ann Surg Oncol (2011) 18:2210–7. doi: 10.1245/s10434-011-1585-7 21308485

[10] Evidence-based practice guidelines for standardized pathological diagnosis of primary liver cancer in China: 2015. Zhonghua Gan Zang Bing Za Zhi (2015) 23:321–7. doi: 10.13315/j.cnki.cjcep.2015.03.001 PMC1277022326427066

[11] RheeHKimHParkYN. Clinico-radio-pathological and molecular features of hepatocellular carcinomas with keratin 19 expression. Liver Cancer (2020) 9:663–81. doi: 10.1159/000510522 PMC776813233442539

[12] ShuyaoWMingyangBFeifeiMXiaoqinH. CK19 predicts recurrence and prognosis of HBV positive HCC. J Gastrointest Surg (2022) 26:341–51. doi: 10.1007/s11605-021-05107-w 34506016

[13] SunDZhangYSunXChenYQiuWJiM. Prognostic value of cytokeratin 19 in hepatocellular carcinoma: A meta-analysis. Clin Chim Acta (2015) 448:161–9. doi: 10.1016/j.cca.2015.06.027 26164382

[14] ZhuoJ-YLuDTanW-YZhengS-SShenY-QXuX. CK19-positive hepatocellular carcinoma is a characteristic subtype. J Cancer (2020) 11:5069–77. doi: 10.7150/jca.44697 PMC737891832742454

[15] HuangXLongLWeiJLiYXiaYZuoP. Radiomics for diagnosis of dual-phenotype hepatocellular carcinoma using Gd-EOB-DTPA-enhanced MRI and patient prognosis. J Cancer Res Clin Oncol (2019) 145:2995–3003. doi: 10.1007/s00432-019-03062-3 31664520 PMC6861194

[16] WuQYuYZhangTZhuWFanYWangX. Preoperative diagnosis of dual-phenotype hepatocellular carcinoma using enhanced MRI radiomics models. Magnetic Resonance Imaging (2022) 57:1185–96. doi: 10.1002/jmri.28391. jmri.28391.36190656

[17] PanJSongMYangLZhaoYZhuYWangM. The role of enhancing capsule and modified capsule appearances in LI-RADS for diagnosing HCC ≤ 3.0 cm on gadoxetate disodium-enhanced MRI. Eur Radiol (2023) 33:5801–11. doi: 10.1007/s00330-023-09487-2 36894754

[18] IshigamiKYoshimitsuKNishiharaYIrieHAsayamaYTajimaT. Hepatocellular carcinoma with a pseudocapsule on gadolinium-enhanced MR images: correlation with histopathologic findings. Radiology (2009) 250:435–43. doi: 10.1148/radiol.2501071702 19095782

[19] LuDSSiripongsakunSKyong LeeJWeiSHChengPMSabounchiS. Complete tumor encapsulation on magnetic resonance imaging: a potentially useful imaging biomarker for better survival in solitary large hepatocellular carcinoma. Liver Transpl (2013) 19:283–91. doi: 10.1002/lt.23597 23280814

The article "Dual-phenotype hepatocellular carcinoma: correlation of MRI features with other primary hepatocellular carcinoma and differential diagnosis" was retracted in 2024. Reason: duplicate publication.

[20] IguchiTAishimaSSanefujiKFujitaNSugimachiKGionT. Both fibrous capsule formation and extracapsular penetration are powerful predictors of poor survival in human hepatocellular carcinoma: a histological assessment of 365 patients in Japan. Ann Surg Oncol (2009) 16:2539–46. doi: 10.1245/s10434-009-0453-1 19533247

[21] PéportéARJSommerWHNikolaouKReiserMFZechCJ. Imaging features of intrahepatic cholangiocarcinoma in Gd-EOB-DTPA-enhanced MRI. Eur J Radiol (2013) 82:e101–106. doi: 10.1016/j.ejrad.2012.10.010 23159401

[22] KimRLeeJMShinC-ILeeESYoonJHJooI. Differentiation of intrahepatic mass-forming cholangiocarcinoma from hepatocellular carcinoma on gadoxetic acid-enhanced liver MR imaging. Eur Radiol (2016) 26:1808–17. doi: 10.1007/s00330-015-4005-8 26373763

[23] AishimaSNishiharaYKurodaYTaguchiKIguchiTTaketomiA. Histologic characteristics and prognostic significance in small hepatocellular carcinoma with biliary differentiation: subdivision and comparison with ordinary hepatocellular carcinoma. Am J Surg Pathol (2007) 31:783–91. doi: 10.1097/01.pas.0000213421.53750.0a 17460464

[24] ZhangLZhouHZhangXDingZXuJ. A radiomics nomogram for predicting cytokeratin 19-positive hepatocellular carcinoma: a two-center study. Front Oncol (2023) 13:1174069. doi: 10.3389/fonc.2023.1174069 37182122 PMC10174303

[25] WangWGuDWeiJDingYYangLZhuK. A radiomics-based biomarker for cytokeratin 19 status of hepatocellular carcinoma with gadoxetic acid–enhanced MRI. Eur Radiol (2020) 30:3004–14. doi: 10.1007/s00330-019-06585-y 32002645

[26] WangHYangCZengMRaoSJiYWengX. Magnetic resonance texture analysis for the identification of cytokeratin 19-positive hepatocellular carcinoma. Eur J Radiol (2019) 117:164–70. doi: 10.1016/j.ejrad.2019.06.016 31307643

[27] NiTShangX-SWangW-THuX-XZengM-SRaoS-X. Different MR features for differentiation of intrahepatic mass-forming cholangiocarcinoma from hepatocellular carcinoma according to tumor size. Br J Radiol (2018) 91:20180017. doi: 10.1259/bjr.20180017 29791202 PMC6209488

[28] ParkHJKimYKParkMJLeeWJ. Small intrahepatic mass-forming cholangiocarcinoma: target sign on diffusion-weighted imaging for differentiation from hepatocellular carcinoma. Abdom Imaging (2013) 38:793–801. doi: 10.1007/s00261-012-9943-x 22829097

[29] WuQYuYXFanYFHuSYaoFRWangXM. The prediction value of enhanced magnetic resonance imaging nomogram model for dual phenotype hepatocellular carcinoma. Zhonghua Yi Xue Za Zhi (2022) 102:1086–92. doi: 10.3760/cma.j.cn112137-20211030-02406 35436807

